# Biomedical Image Classification in a Big Data Architecture Using Machine Learning Algorithms

**DOI:** 10.1155/2021/9998819

**Published:** 2021-05-30

**Authors:** Christian Tchito Tchapga, Thomas Attia Mih, Aurelle Tchagna Kouanou, Theophile Fozin Fonzin, Platini Kuetche Fogang, Brice Anicet Mezatio, Daniel Tchiotsop

**Affiliations:** ^1^College of Technology, University of Buea, Buea, Cameroon; ^2^Department of Research, Development,Innovation and Training, InchTech's, Yaoundé, Cameroon; ^3^Department of Electrical and Electronic Engineering, Faculty of Engineering and Technology (FET), University of Buea, P.O. Box 63, Buea, Cameroon; ^4^Research Unity of Condensed Matter, Electronics and Signal Processing, Department of Physics, Faculty of Science, University of Dschang, P.O. Box 67, Dschang, Cameroon; ^5^Research Unity of ‘Automatic and Applied Informatic,IUT-FV of Bandjoun, University of Dschang-Cameroun, B.P. 134 Bandjoun, Dschang, Cameroon

## Abstract

In modern-day medicine, medical imaging has undergone immense advancements and can capture several biomedical images from patients. In the wake of this, to assist medical specialists, these images can be used and trained in an intelligent system in order to aid the determination of the different diseases that can be identified from analyzing these images. Classification plays an important role in this regard; it enhances the grouping of these images into categories of diseases and optimizes the next step of a computer-aided diagnosis system. The concept of classification in machine learning deals with the problem of identifying to which set of categories a new population belongs. When category membership is known, the classification is done on the basis of a training set of data containing observations. The goal of this paper is to perform a survey of classification algorithms for biomedical images. The paper then describes how these algorithms can be applied to a big data architecture by using the Spark framework. This paper further proposes the classification workflow based on the observed optimal algorithms, Support Vector Machine and Deep Learning as drawn from the literature. The algorithm for the feature extraction step during the classification process is presented and can be customized in all other steps of the proposed classification workflow.

## 1. Introduction

The healthcare field has experienced rapid growth in medical data in recent years. In 2018, the USA generated a zettabyte of healthcare data [1]. In the wake of this agglomeration of medical data, especially images, the use of new methods based on big data technologies, machine learning (ML), and artificial intelligence (AI) has therefore become necessary. Big data is generally identified by five major characteristics called the “5V”: volume (amount of data generated), variety (data from different categories), velocity (speed of data generation), variability (inconsistency of data), and veracity (quality of captured data) [1–8]. The application of information technologies to the healthcare field raises opportunities for the development of new diagnostics and treatments, making it a critical area of investigation. The new ideas, concepts, and technologies based on big data, ML, and AI are proposed to improve the healthcare field. Nowadays, many works are performed to use big data to manage and analyze healthcare systems. El aboudi and Behlima proposed a big data management approach for healthcare systems [9]; Tchagna et al. proposed a complete big data workflow for biomedical image analysis [7]; Belle et al. showed the impact of big data analysis in healthcare [10]; Luo et al. in [2] performed a literature review of big data application in biomedical research and healthcare; Viceconti et al., as far as they are concerned, examined the possibility of using big data for personalized healthcare [11]; Archenaa and Anita in 2015 showed the need for big data analytics in healthcare to improve the quality of healthcare as follows: providing patient-centric services, detecting spreading diseases earlier, monitoring the hospital's quality, and improving the treatment methods [12]. Thus, when big data technologies are incorporated into a framework or applications, better data handling and higher performance can be achieved [13]. Based on those works, it was noticed that the biomedical system is converging to a big data platform that presents us with an opportunity to efficiently manage and analyze this huge and growing amount of biomedical data.

A vast quantity of data in healthcare constitutes data images captured from medical imaging (Computed Tomography Scan, Echography, Mammography, MRI, etc.). To achieve complete management and analysis of biomedical images, we have to automate all steps proposed in [7]. One of the most necessary steps is classification. Classification in ML concerns a problem of identifying to which set of categories a new population belongs [7]. A good classification performed essentially leads to a good automatic diagnosis of diseases on an image. This is in order that the diagnostic algorithms can adapt accordingly to the image groups resulting from the classification. So, classification is an important step in a biomedical automatic system.

In a new concept for biomedical images analysis using big data architecture proposed in 2018 by Tchagna et al. in [7], the authors present a workflow performing the steps of acquisition of biomedical image data, analysis, storage, processing, querying, classification, and automatic diagnosis of biomedical images. The workflow was performed with unstructured and structured image data based on a NoSQL database. The authors proposed a Spark architecture that allows developing appropriate and efficient methods to leverage a large number of images for classification. However, in their work, they did not explain very well the algorithm used for biomedical image classification. Based on this gap, the paradigm in this paper is to present and discuss methods and algorithms used to perform a good classification for the biomedical image in big data architecture.

This paper specifically focuses on biomedical imaging with big data technologies along with ML for classification. It presents a set of algorithms that can be used to accomplish the classification step in big data architecture. It further describes the importance of applying the classification of biomedical images in big data architecture. Based on the Spark framework, this work proposes an algorithm to perform the steps of the proposed classification workflow. ML plays an important role in biomedical image classification, and when combined with big data technologies, the processing is done with less time and can handle a lot of images at the same time. The rest of this paper is organized as follows.  Section 2 reviews published methods in the field. In Section 3, these methods are explored theoretically throughout our work.  Section 4 presents the Spark algorithm. A conclusion and future work are provided in Section 5.

## 2. A Survey of Biomedical Image Classification Methods

The healthcare field is distinctively different from other fields. Healthcare is generally delivered by health professionals. Pharmacy, dentistry, nursing, midwifery, medicine, audiology, optometry, occupational therapy, psychology, physical therapy, and other health professions are all part of healthcare. Healthcare is a high-priority field and people expect the highest level of care and services. It is most difficult for specialists to identify complex disease patterns from large amounts of images. Hence, each specialist will be limited to visualizing only the biomedical images essentially related to his field of competence, which is somewhat restrictive. In contrast, ML, deep learning (DL), and AI excel at automatic pattern recognition from large amounts of biomedical image data. In particular, machine learning and deep learning algorithms (e.g., support vector machine, neural network, and convolutional neural network) have achieved impressive results in biomedical image classification [14–23]. Classification helps to organize biomedical image databases into image categories before diagnostics [24–30]. Many investigations have been performed by researchers to improve classification for biomedical images [6, 7, 31–36]. In 2016, Miranda et al. surveyed medical image classification techniques. They reviewed the state-of-the-art image classification techniques to diagnose human body disease and covered identification of medical image classification techniques, image modalities used, the dataset, and tradeoff for each technique [31]. They concluded that artificial neural network (ANNs) classifier and SVM are the most used technique for image classification because these techniques give high accuracy, high sensitivity, high specificity, and high classification performance results [31]. In the same logic, Jiang et al. in 2017 made an investigation on ML algorithms for healthcare [32]. They grouped algorithms by the category of ML (Supervised, Unsupervised, and Semisupervised) and provided a graphical representation. Supervised learning algorithms are used for classification. They showed that SVM and ANNs are two famous algorithms used to classify biomedical image data. In medical imaging, SVM and ANN take up to 42% and 31%, respectively, of the most used algorithms [32]. Similarly, Wang et al. in [6] confirmed that the SVMs and ANNs are good classifiers.

In 2007, Jiang et al. used the Rough Set Theory (RTS) to improve SVM for classifying digital mammography images [33]. They reported 96.56% accuracy. However, their work is only limited to mammography images, and they used structured data. But in reality, the vast majority of images' data come from many sources that are unstructured. Jeved et al. proposed in [34] a technique to classify brain images from Magnetic Resonance Imaging (MRI) using perceptual texture features, fuzzy weighting, and support vector machine. Their proposed technique classifies normal and different classes of abnormal images, and they used fuzzy logic to assign weights to different feature values based on its discrimination capability. Lu and Wang in 2012 applied the SVM to breast multispectral magnetic resonance images to classify the tissues of the breast. They compared their method with the commonly used C-means for performance evaluation and proved that the SVM is a promising and effective spectral technique for MR image classification [35]. Although the two methods majorly mentioned above are efficient, their applications in image classification are limited only to a few kinds of medical images. Deep learning comes with many hidden networks to improve the efficiency of classification performance when the datasets are very large. For this reason, khan et al. in [36] proposed a modified convolutional neural network (CNN) architecture for automatically classifying anatomies in medical images by learning features at multiple levels of abstractions from the data obtained. They also provided an insight into the deep features that have been learned through training, which will help in analyzing various abstraction of features ranging from low level to high level and their role in the final classification, and obtained a test accuracy of 81% [36]. Li et al. in [37] proposed a customized CNN network for lung image patch classification and designed a fully automatic neural-based machine learning framework to extract discriminative features from training samples and perform classification at the same time. They showed that the same CNN architecture can be generalized to perform other medical image or texture classification tasks. In 2018, Ker et al. discussed the DL applications in medical image classification, localization, detection, segmentation, and registration [38]. They focused on CNN and explained all methods to perform each task. Concerning classification, they gave examples of disease classification tasks by using CNN. In 2020, Zhang et al. looked for how to accelerate the processes of learning time with large-scale multilabel image classification using the CNN method for learning and building the classifier with an unknown novel group that came in a stream during the training stage [39]. However, their classifier/model is essentially on the ability of the novel-class detector that can give the worse result when multiple novel classes may exist. Vieira et al. provided a review of the studies of applying DL to neuroimaging data to investigate neurological disorders and psychiatric. They compare the different ML algorithms with DL algorithm in neuroimaging and show that DL gives good results compared to ML such as SVM when the dataset is important [40]. Nalepa and Kawulok in 2019 performed an extensive survey on existing techniques and methods to select SVM training data from large datasets and concluded that the DL will be more efficient than SVM for large datasets [41]. Badar et al. show how to apply DL in Retina image classification and identification to detect diseases such as diabetic retinopathy, macular bunker, age-related macular degeneration, retinal detachment, retinoblastoma, and retinitis pigmentosa [42]. Yan et al. in 2019 proposed a novel hybrid CNN and RNN for breast cancer image classification by using the richer multilevel feature representation of the histopathological biomedical image patches [43]. Zareapoor et al. used a combination of DL and a nonlinear-SVM to deal with extremely large datasets to improve the learning time of their model. However, the learning time remains and DL is today a problem with their model [44]. Fang et al. proposed a CNN architecture method for breast cancer classification by constructing a multi-SVM-based biomedical image kernel using quality scores got to achieve the classification [45]. Kotsiantis in [46] compares the features of learning techniques for classification.  Table 1 shows the summary of this comparison. As Jiang et al. in [32], they concluded that the SVM and ANNs are the best algorithms used for classification problem in biomedical image. However, they established this conclusion when the amount of data is not large. So today, we can replace ANNs with CNN when we work on a large dataset.

Based on the previously cited literature in this section, it was observed that the classifier algorithms depend on the amount of data of images in the input of the classification system. For example, for a medium dataset, SVM outperforms another classification algorithm like DL. Indeed, the SVM classifier often outperforms many commonly used ML algorithms, even though it may not be an ideal choice to handle large datasets [47–51]. For a large dataset, DL outperforms another classification algorithm [23, 39, 52–55]. Despite the notable advantages of DL and SVM, challenges in applying them to the biomedical domain still remain. It was noticed that none of these works have made their classification with big data tools. Indeed, classification can be performed with big data technologies for these reasons:

1. In order to swiftly work with both unstructured and structured biomedical images (inferring knowledge from complex heterogeneous patient data/leveraging the patient data image correlations in longitudinal records)
2. Rapid queries and access to biomedical images database
3. Prospect of a database based on NoSQL technologies
4. Personalized classification algorithm to the patient
5. Opportunity to efficiently handle massive amounts of biomedical image data
6. Easy to analyze data images using machine learning and artificial intelligence
7. Implementation of the MapReduce programming (parallel programming) in those frameworks (Hadoop, Spark)

Furthermore, in the previously cited works in this section, the authors did not show what is the impact of big data in their works, if any. This drawback is one of the main interests of this paper. This paper, therefore, presents a designed workflow for biomedical image classification based on SVM and DL (CNN), which could be implanted in big data architecture.

## 3. System Classification Workflow for Biomedical Images

The application of ML technology with SVM, especially DL with CNN, to biomedical image classification field research has become more and more popular recently. The main objective of medical image classification is to identify which parts of the human body are infected by the disease and not only to reach high accuracy. In the proposed workflow, according to the previous section, there are two algorithms to perform classification with good accuracy: one for a medium dataset and the other for a large-scale dataset. SVM and DL are then used, respectively, in this regard. The classification processes are as depicted in Figure 1.

In Figure 1, the system workflow to perform a biomedical image classification is presented. As shown in the workflow, the classification process is performed in two basic steps. In the first step, a classifier model is built based on the labeled biomedical image using ML (SVM or CNN) algorithms. When the classifier model has been derived, any unlabeled biomedical images can be presented to the model in order to make predictions about the group to which such images belong.  Figure 2 presents a DL along with CNN architecture for image classification. The following section presents how we deal with training and testing datasets in classification.

### 3.1. The Training Phase

The first part of Figure 1 is the training phase. The training phase in classification concerns the phase where you present your data from the training dataset (labeled biomedical images in this case), extract features, and train your model, by mapping the input with the expected output. Here, the network can learn by using a Gradient Descent Algorithm (GDA). The purpose of GDA is to find the different values of the network weights that best minimize the error between the true and estimated outputs [56–59]. Backpropagation is the name of this propagation procedure and permits the network to predict how much the weights from the lower layers network have to be changed by the GDA. The training phase has traditionally three main steps: labeled biomedical image dataset retrieval, feature extraction, and machine learning algorithm (SVM or CNN).

#### 3.1.1. Labelled Biomedical Image

In general, labeled images (training dataset) are used to perform the machine learning of the class (group) description which in turn is used for unknown (unlabeled) images [60]. Since the supervised learning paradigm is adopted in this workflow, the labeled biomedical images dataset is the most suitable for the learning phase in this workflow.

#### 3.1.2. Feature Extraction

An image is represented by a set of descriptors that structure the feature vectors and is formed by pixels, which may or may not represent features. A feature is defined as an interesting part of an image and is used as a starting point for computer vision algorithms [61]. When the features are extracted from a labeled biomedical image dataset, classification is then done using a classification method such as SVM or DL. When the classification is performed by using DL, the features are called deep features.

#### 3.1.3. Machine Learning Algorithm (SVM or CNN)

The support vector machine (SVM) is a supervised learning method that generates input-output mapping functions from a set of labeled training data [62]. Originally, SVM is a binary classifier that works by identifying the optimal hyperplane and correctly divides the data points into two classes [63]. There will be an infinite number of hyperplanes and SVM will select the hyperplane with maximum margin. The margin indicates the distance between the classifier and the training points (support vector) [63, 64]. SVM is mainly used to deal with classification and regression problems. There are three steps of the SVM algorithm, Identification of Hyperplane, classification of classes, and finding hyperplane to separate classes [64, 65]. The training principle behind SVM is to find the optimal linear hyperplane so that the expected classification error for unseen test samples should be minimized [34, 60]. SVM is a margin-based classifier that achieves superior classification performance compared to other algorithms when the amount of dataset training is medium [34, 51, 60].

DL techniques are conquering the prevailing traditional approaches of the neural network; when it comes to the huge amount of dataset, applications requiring complex functions demanding increase accuracy with lower time complexities [22, 66, 67]. DL particularly CNN has shown an intrinsic ability to automatically extract the high-level representations from big data [36]. CNN is an artificial neural network with many hidden layers of units between the input and output layers and millions or billions of parameters [21, 68–71]. General, DL architecture is composed of one or more convolutional layers with many hidden networks, one or more max pooling operations, and a full connection layer. This feeds into a final Fully Connected Layer which assigns class scores or probabilities, thus classifying the input into the class with the highest probability [38]. To apply a CNN on an image, we have this image in the input to the network. The network has an input layer that takes this image as the input, an output layer from where we obtain the trained output, and the intermediate layers called the hidden layers. The network has a series of subsampling and convolutional layers. The layers produce together an approximation of input image data. DL is very good at learning the local and global structures from image data [37]. However, the CNN exploits spatially local correlation by enforcing a local connectivity pattern between neurons of adjacent layers [72]. Deep learning enables the extraction of multiple feature levels from data directly without explicit definition. It provides a higher level of feature abstraction, thus potentially providing better prediction performance [73, 74]. Research works based on CNN significantly improved the best performance for many image databases [37, 75]. So, to apply DL, the dataset of the image has to contain many images.

### 3.2. Testing Phase

In the testing phase, the feature vectors of the unlabeled biomedical image dataset serve as input. A classifier decided on the basis of the classifier model, with its own classification rules, to which class/group that feature vector belongs. The testing phase has four main steps: unlabeled biomedical image capturing, feature extraction, classifier model, and prediction. The feature extraction step in the testing phase is performed as in the training phase.

#### 3.2.1. Unlabeled Biomedical Image

The unlabeled biomedical images dataset is used to provide an unbiased evaluation of a final model fit on the labeled biomedical images dataset.

#### 3.2.2. Classifier

A classifier is trained on the extracted features. The goal of a classifier is to distinguish images of the known class from images of alien classes. Thus, a classifier is required to learn so that it can identify out-of-class (alien) images. The SVM and DL classifiers are used to perform verification for the next stage of prediction.

#### 3.2.3. Prediction

Based on SVM or DL classifier, the prediction stage in the workflow allows predicting automatically into which class an image belongs. Here, we can evaluate the prediction average accuracy for both SVM and DL. However, as drawn from the literature, it is established that for a large dataset, the accuracy of the DL classifier is generally better than the SVM classifier. And for a medium dataset, the classifier of SVM is better than the DL classifier.

One of the characteristics of big data is the volume (amount of data generated). To apply the classification workflow of Figure 1 in big data architecture, we have to verify this rule for the dataset that is presented to the workflow's training phase. However, taking into consideration the size of the dataset we can perform classification on, we can use SVM or DL as explained in the previous subsection. Here, the performance of the network can be evaluated by several performance parameters such as sensitivity, accuracy, specificity, and F-score. Sensitivity refers to the proportion of true positives correctly identified, specificity refers to true negatives correctly identified, and the accuracy of a classifier/model represents the overall proportion of correct classifications [58, 59]. Spark framework is one of the best frameworks used to perform big data processing. In the next section, an algorithm to perform some stages of Figure 1 is presented, based on the Spark framework of image classification in [7].

## 4. Spark Algorithm for Biomedical Image Classification

Apache Spark is a distributed computing platform used in the big data scenario that has become one of the most powerful frameworks. Spark offers a unified and complete framework to manage the different requirements for big data processing with a variety of datasets (graph data, image/video, text data, etc.) from different sources (batch, real-time streaming) [7]. Spark framework has been created to overcome the problems of the Hadoop framework according to its creators. Indeed, the Spark framework has proved to perform faster than Hadoop in many situations (more than 100 times in memory). With capabilities like in-memory data storage and near real-time processing, the performance can be several times faster than other big data technologies. Spark framework is able to make data suitable for iteration, query it repeatedly, and load it into memory. In the Spark framework, the main program (driver) controls multiple slaves (workers) and collects results from them, whereas slaves' nodes read data partitions (blocks) from a distributed file system execute some computations and save the result to disk. Spark as Hadoop is based on parallel processing MapReduce that aims at automatically processing data in an easy and transparent way through a cluster of computers. In addition to Map and Reduce operations, Spark also supports SQL queries, streaming data, machine learning, and graph processing data [7]. In Spark, sometimes, we can program and execute our algorithm on many clusters at the same time. For instance, Figure 3 shows the links between four nodes to perform data processing.

Figure 3 shows the possibility of the processing of data in four nodes, where the master node and the slave nodes are defined. The master manages and distributes the job to the slave. According to the volume of the dataset, you can choose more or less than three slaves. The number of slaves leads to the gaining of processing time.

In Spark DataFrame, the importation and representation of images follow the pipeline as shown in Figure 4.

This pipeline consists typically of the image import, preprocessing, model training, and inferencing stages.

In this section, we propose a Spark algorithm to perform some stages of Figure 1. Image feature is an image pattern, based on which we can describe the image with what we see. The main role of features in image biomedical classification is to transform visual information into vector space. Thus, we can perform mathematical operations on them and find similar vectors. To perform feature selection, the first issue is to detect features on a biomedical image. The number of them can be different depending on the image, so we add some clauses to make our feature vector always have the same size. Then, we build vector descriptors based on our features; each descriptor has the same size. It should be noted that there are different approaches to write this Spark algorithm for each step of Figure 1.  Algorithm 1 presents a method to perform feature extraction by using Spark framework with its MapReduce programming. In this algorithm, it should be noted that the feature extraction from the unlabeled or labeled image is performed with many images in the big data context with respect to the different V of big data (volume, velocity, variety, variability, and veracity). However, the performances of the Spark framework can be decreased in some situations: especially during the feature extraction, in a situation where there are some small images in the dataset (unlabeled biomedical images/labeled biomedical images). Another instance is if the size of the image considered is too different from one another, it will cause an unbalanced loading in the Spark. To solve these problems, in [76], the authors introduced two methods: sequence in feature extraction and feature extraction by segmentation. The implementation of one of these two methods can resolve the problem of unbalanced loading and the running time of each job can also be the same.

The process of classification is a function that is started when new unlabeled data comes to the system.  Algorithm 2 predicts the image's class by identifying to which set of categories this image belongs. In the algorithm, both prediction and query are performed in the same **MapReduce** phase.

By adopting the Spark framework, there comes an advantage to work in a big data environment and use its embedded libraries like MLlib (Machine Learning libraries).

## 5. Comparison of Machine Learning Methods and Applications' Use in the Literature

To perform this comparison, we are based on some works done in the literature.  Table 2 gives us an overview of different works done in the literature in ML with their application.

Table 2 helps us to see that ML algorithms are very used in biomedical application and today in a lot of applications also. Many researches as Wang et al., Tchagna Kouanou et al., or Chowdharya et al. performed a good job and published a lot of papers in this exciting domain.

We can also conclude that, nowadays, as the size of the training data set grows, ML algorithms become more effective. Therefore, when combining big data technologies with ML, we will benefit twice: these algorithms can help us keep up with the influx of data, and the amount and variety of the same data can help and grow the algorithms. ML and big data are the current blue chips in the IT industry. The storage of big data technologies analyzes and extracts information from a large amount of data. On the other hand, ML is the ability to learn and improve automatically from experience without explicit programming [7].

## 6. Conclusion

In this paper, we have focused on the concept of big data for biomedical image classification tasks and, in particular, on exploring machine learning algorithms (SVM and DL) for biomedical classification following the Spark programming model. We have proposed a workflow with essential steps for biomedical image classification. Based on the literature surveyed, the SVM and DL were found to be the two possible candidate algorithms that can be used to perform biomedical image classification. In the survey, it was established from the literature that SVM gives a good performance when the size of the dataset is medium while the DL is established to have good performance when the dataset is of large scale. Therefore, we can choose which machine learning algorithm to use for classification based on the size of the dataset at hand. Spark is the framework that we proposed for the implementation of the proposed workflow. We have given a Spark algorithm to perform feature extraction in our proposed workflow. It should be noted that this algorithm can be customized and applies to another step. As future work, we propose to make a real-world implementation of our Spark algorithm and calculate all performance parameters as in [77–79], where the authors implemented the algorithm for image compression that we can use in the workflow proposed in [7].

## Figures and Tables

**Figure 1:** Classification system workflow for training and testing processes.

**Figure 2:** Convolutional neural network (CNN) architecture for biomedical image classification.

**Figure 3:** Job execution Apache Spark in four clusters: one master and three slaves.

**Figure 4:** Importing images in Spark DataFrame.

**Algorithm 1:** Feature extraction process.

**Algorithm 2:** Prediction process.

**Table 1:** Comparison of classification methods in biomedical image based on the literature [32, 46].

	Decision trees	Neural networks	Naïve bayes	KNN	SVM	Rule-learning
Accuracy	∗∗	∗∗∗	∗	∗∗	∗∗∗∗	∗∗
Speed of classification	∗∗∗∗	∗∗∗∗	∗∗∗∗	∗	∗∗∗∗	∗∗∗∗
Tolerance to redundant attributes	∗∗	∗∗	∗	∗∗	∗∗∗	∗∗
Speed of learning	∗∗∗	∗	∗∗∗∗	∗∗∗∗	∗	∗∗
Tolerance to missing values	∗∗∗	∗	∗∗∗∗	∗	∗∗	∗∗
Tolerance to highly interdependent attributes	∗∗	∗∗∗	∗	∗	∗∗∗	∗∗
Dealing with discrete/binary/continues attributes	∗∗∗∗	∗∗∗ (not discrete)	∗∗∗ (not continuous)	∗∗∗ (not directly discrete)	∗∗ (Not discrete)	∗∗∗ (not directly discrete)
Tolerance to noise	∗∗	∗∗	∗∗∗	∗	∗∗	∗
Dealing with a danger of overfitting	∗∗	∗	∗∗∗	∗∗∗	∗∗	∗∗
Attempts for incremental learning	∗∗	∗∗∗	∗∗∗∗	∗∗∗∗	∗∗	∗

^∗∗∗∗^Very good. ^∗∗∗^Good. ^∗∗^Fairly Good. ^∗^Bad.

**Table 2:** Some ML methods and application comparison.

Authors	Deep learning methods	Machine learning method	Big data technologies	Applications
Luo et al. [2]	No	No	Yes (Hadoop)	Healthcare
Tchagna Kouanou et al. [7]	No	No	Yes (Spark and Hadoop)	Biomedical images
Manogaran and Lopez [8]	No	Yes	Yes	Healthcare
Thrall et al. [17]	No	Yes	No	Radiology
Fujiyoshi et al. [24]	Yes	No	No	Image recognition
Tchagna Kouanou et al. [77]	No	Yes (K-Means- unsupervised learning)	No	Biomedical image compression
Tchagna Kouanou et al. [78]	No	Yes (K-Means- unsupervised learning)	Yes (Hadoop)	Biomedical image compression
Tchagna Kouanou et al. [79]	No	Yes (K-Means- unsupervised learning)	No	Image compression
Alla Takam et al. [80]	Yes (CNN)	No	Yes (Spark)	Biomedical image
Chowdhary and Acharjya [81]	No	Yes (fuzzy C-means)	No	Feature extraction and segmentation
Bhattacharya et al. [82]	Yes	No	No	Biomedical image
Chowdhary et al. [83]	Yes	No	No	Biomedical images (breast cancer classification)
Wang et al. [84]	Yes (CNN, hierarchical loss)	No	No	Biomedical images (breast cancer classification)
